# Hybrid Model for Detection of Cervical Cancer Using Causal Analysis and Machine Learning Techniques

**DOI:** 10.1155/2022/4688327

**Published:** 2022-05-04

**Authors:** Umesh Kumar Lilhore, M. Poongodi, Amandeep Kaur, Sarita Simaiya, Abeer D. Algarni, Hela Elmannai, V. Vijayakumar, Godwin Brown Tunze, Mounir Hamdi

**Affiliations:** ^1^KIET Group of Institutions, Delhi-NCR, 201206, India; ^2^Division of Information and Computing Technology, College of Science and Engineering, Hamad Bin Khalifa University, Qatar Foundation, Doha, Qatar; ^3^Chitkara University Institute of Engineering and Technology, Chitkara University, Punjab, India; ^4^Department of Information Technology, College of Computer and Information Sciences, Princess Nourah bint Abdulrahman University, P.O. Box 84428, Riyadh 11671, Saudi Arabia; ^5^University of New South Wales, Sydney, Australia; ^6^Department of Electronics and Telecommunication Engineering, Mbeya University of Science and Technology, Mbeya, Tanzania

## Abstract

Cervical cancer has become the third most common form of cancer in the in-universe, after the widespread breast cancer. Human papillomavirus risk of infection is linked to the majority of cancer cases. Preventive care, the most expensive way of fighting cancer, can protect about 37% of cancer cases. The Pap smear examination is a standard screening procedure for the initial screening of cervical cancer. However, this manual test procedure generates many false-positive outcomes due to individual errors. Various researchers have extensively investigated machine learning (ML) methods for classifying cervical Pap cells to enhance manual testing. The random forest method is the most popular method for anticipating features from a high-dimensional cancer image dataset. However, the random forest method can get too slow and inefficient for real-time forecasts when too many decision trees are used. This research proposed an efficient feature selection and prediction model for cervical cancer datasets using Boruta analysis and SVM method to deal with this challenge. A Boruta analysis method is used. It is improved from of random forest method and mainly discovers feature subsets from the data source that are significant to assigned classification activity. The proposed model's primary aim is to determine the importance of cervical cancer screening factors for classifying high-risk patients depending on the findings. This research work analyses cervical cancer and various risk factors to help detect cervical cancer. The proposed model Boruta with SVM and various popular ML models are implemented using Python and various performance measuring parameters, i.e., accuracy, precision, *F*1–Score, and recall. However, the proposed Boruta analysis with SVM performs outstanding over existing methods.

## 1. Introduction

According to a WHO survey, cervical cancer has probably led to cause cancer affecting women in underdeveloped nations [1]. Despite medical centers, there have been thousands of new cases within the USA in 2016, compared to more than 20K morality in 2014. This cervical cancer database comprises more than 800 data sample values, 32 characteristics, and four objectives, which have been reported in the year 2016-17. Essential features include aggregate characteristics, tobacco behaviors, and health records from the past. The several testing and diagnostic procedures that result in an excellent diversity add to the data's complication. As a result, the vital issue involves predicting the person's component behavior and determining the optimum screening technique. As a result, the fundamental problem in predicting the person's component risk assessment is the process of the optimum main channel. Various investigators have examined cervical cancer data collected from different sources [2]. The primary risk factors for cervical cancer transmission are poor menstruation sanitation, adolescent pregnancy, cigarettes, and oral prevention methods. Healthcare datasets have more characteristics and incomplete data than nonmedical datasets. By form of enhancement, it is essential to define the significant and necessary attributes for quantitative model construction. ML techniques are superior in forecasts and performance tuning expeditions, but they have been widely used in cancer and breast cancer research [3]. According to a study [4], long-term HPV infectious disease is the primary cause of cervical cancer.

On the other hand, if diagnosed early and cured correctly, cervical cancer is the most curable type. The technique mentioned above requires more effort to process the information, and obtained low-level features cannot deliver optimal classification efficiency, highlighting the failures of intelligent learning. An ML-based feature extraction approach shares massive advantages over all other cancer detection algorithms in obtaining an improved CAD framework. The ML-based technique accomplishes state-of-the-art findings on complicated computer vision applications [5]. As per existing studies, most cervical precancerous disease classification investigations focus on individual colposcopy visualizations during acetic acid tests, making it challenging to determine cervical cancer. This article focuses on numerous machine learning techniques that can forecast the occurrence of cervical cancer as precisely as feasible, utilizing a fixed number of factors of potential risk determinants for each female. However, the stability of recall and precision is a challenging issue once working to develop a forecasting model with a set of analyses. This research presents a prediction model using machine learning methods to detect cervical cancer analysis. This research proposed an efficient feature selection and prediction model for cervical cancer datasets using Boruta analysis and SVM method to deal with this challenge. This research utilized SVM, random forest, decision tree, and Boruta methods to analyze the cervical cancer dataset. This strongly supports feature classification, regression, clustering, and survival analysis with more modeling methods.

The research work [6] involves the identification of accurate indicators from the UCI dataset that can act as powerful predictors of cervical cancer and a dependent variable that may be a function of these predictions for visualizing and analysis of the cancer trends. Multiple models may be built to find the indicators that can help understand the dynamics of the various variables. The performance of the proposed model and existing ML model is verified using an online cervical cancer dataset using Python and different version measuring parameters, i.e., accuracy, precision, *F*1 score, and recall. This research is aimed at developing mathematical equations and applying Boruta analysis to depict two types of cervical cancers: (a) low-risk and (b) high-risk cancer. First of all, the cervical cancer dataset has been identified, and the preprocessing has been performed on the dataset, followed by correlation analysis and Boruta analysis. After this, causal analysis has been done that helps identify factors that contribute to cervical cancer. The workflow includes making hypotheses that will be further verified and validated by the results.

The complete research work is organized as follows: Section 1 covers the cancer-related introduction work.  Section 2 covers the review of existing research and also suggested a comparative analysis of various methods for cancer research. Similarly, Section 3 covers the materials and techniques, Section 4 covers experiments and results analysis, and finally, Section 5 covers the conclusion and future directions of the research.

## 2. Literature Review

This research presents a machine learning method-based model for earlier cervical cancer prediction in the early stage. This section represents the review of various machine learning models for earlier and more accurately cervical cancer detection. The review work is divided into three subsections based on the risk factor, a mathematical model, and machine learning methods.

### 2.1. Based on Risk Factors for Cervical Cancer

The “National Comprehensive Cancer Network” has issued a warning about the benefits of initial identification of cervical cancer. In contrast, a postponement in treatment is the leading cause of an increasing number of women mortality globally. As a result, numerous scientific and medical investigations have investigated the causes, symptoms, and methodologies of identifying and avoiding cervical cancer. Researchers have also attempted to evaluate the risks that contribute to the pathogenesis and progression of this particular cancer. The selected research works are as follows.

In the research article [7], the cure for cancer has usually taken numerous forms over the years; total elimination may not even be possible; however, the disease's probability of occurrence and forecasting can be reduced. Any disorder can be healed if identified in its beginning phases, and cancer can be successfully treated if spotted in its beginning phases. On the other hand, cervical cancer is hard to forecast in its early stages because there are no symptomatic. The frequent test is done for such forecasting of cancer cells because testing has been the only way it can be forecasted [8]. In [9], to avoid such uncertainties, screening outcomes may be supervised as false positives at points in time, or they may be postponed. Machine learning has been developed in the field of health care services. Numerous methods, techniques, and technology have been used to anticipate cancer cells quicker and with a lower false-positive rate.

The method of mathematical modeling aids in the comprehension of the observable occurrence. The visible event in the healthcare area [10] could be wellness symptoms and perhaps a sickness, and this technique results in a workable characterization of complicated things. Inside the medical sciences, the mathematical formulation has also been utilized in various methods to solve, reproduce, research, and explain biological mechanisms [11]. The research [12] proposes probabilistically mathematical systems when the sample sizes are limited and can thoroughly examine the parameters. According to the researchers, any healthcare system may comprehend via comparisons; then, such a procedure must influence the mathematical framework [13]. As illustrated, a model named three separate structures might be used to understand the number of carbohydrates stored in human bodies. Other researchers prefer to use informative computational methods. These models use a feasible description of factors in analytics testing to describe realistic circumstances [14]. In social and epidemiology investigations, description methods are essential. In most cases, the means, median, average, standard deviation and variance, and other statistics are determined, and a report of the phenomena is written down.  Table 1 represents the summary of existing research work based on cancer risk factors.

### 2.2. Based on Mathematical Models

Furthermore, more examination into cervical cancer using mathematical models indicates that significant teams of investigators in the medical sciences concentrate on diagnostics modeling models [28]. The experts in clinical forecasting use a variety of strategies to construct models. Analysis technique and supervised learning model are two examples. Specific healthcare computer models are referred to as “forms of modern.” Basic logical reasoning, hypotheses, concepts, and descriptive analysis have created these frameworks. Many researchers usually refer to such algorithms as medical condition recognition systems [29]. They also utilized ML algorithms to predict serious health issues by the researchers. Enzyme kinetics and pharmacokinetics are two necessary fields of medical research [30]. Machine learning algorithms and automatic analyses are frequently used in several areas of medicine. Physiological reactions and parameters like stress levels, heartbeat, and others must be recorded and modeled for tracking medical conditions within time-series modeling techniques [31]. Modeling, which enables to comprehension of dynamic interaction, uses an approach called transferring characteristics for a detailed look. This type of procedure keeps track of feedback and the processes between this. Many researchers have looked at the principal source of such medical conditions while discovering and establishing the mathematical determinant factors.

Nevertheless, the issue is mainly identifying acceptable factors that can describe the specialized clinical paradigm or phenomenon and determining which independent variables may operate as potential forecasters and which characters can describe the entire computational formula [32]. All of the clinical models presented thus far depend on a fundamental grasp of the mathematical model development. Depending on the concerns and obstacles described in the present research, this next section considers the frame of the activity.  Table 2 represents the review of cancer types based on several features and age group impact.

### 2.3. Based on Machine Learning Models

In this research, machine learning techniques have been employed to detect cervical cancer accurately via constructing a framework affected by previous research methods in a similar domain. Research [42] proves that by utilizing the oversampling process performance of existing approaches can be improved. This research used the random forest to build a classifier predicated on cervical cancer cases. The analysis indicates that the RF significantly outperformed its same framework after implementing SMOTE, including all characteristics of cervical disease variables in the forms of parameters, i.e., accuracy, specificity, precision, and true positive rate. The research [43] used the online UCI dataset with various strategies for cervical cancer diagnosis: (a) SVM, (b) SVM with PCA, and (3) SVM with RFE. This article concluded that SVM performs well and achieves better precision, diagnostic accuracy, and precision than the multiple different classifiers.

Research [44] utilized three forms of machine learning models to categorize the UCI cervical cancer data. The proposed model used a “border row hierarchical clustering” (BRHC) to deal with dataset inequity. This research has observed that the XG-Boost and random forest methods perform outstandingly in cancer prediction accuracy rates. Since this cancer data contains many incomplete, missing data, it is necessary to deal with missing attributes carefully. Research [45] offers four distinct methods to deal with missing values in the cancer dataset. These techniques are NOCB, LOCF, FVM, and NOCB. To anticipate the biopsy input variables, they utilized six algorithms: LR, RF, SVM, DT, NB, and NN [46], and researchers also concluded that if used with the NOCB preprocessing phase, the SVM, as well as LR, reached the best accuracy, *F*1 measure, and precision. In this research, machine learning techniques have been employed to detect cervical cancer accurately via constructing a framework affected by previous research methods in a similar domain. The private database was created using 472 survey questions from a China health center, so each cancer patient who took the poll had a correlating gene sequence set of data. This research collects the data from “Mexico's Maggiore de Caracas health center.” This dataset contains 592 cancer patients' data with various attributes. This research applied a pooling and discussed the difficulties associated with conventional cervical cancer diagnostics.  Table 3 represents the comparison of research methods based on ML methods.

Machine learning approaches have been utilized in this investigation to correctly identify cervical cancer via developing a structure influenced by prior research methodologies used in a similar field. The public available UCI dataset on cervical cancer does not have per-annotated rows that give a confirmatory signal about the presence or absence of cervical cancer. The dataset aims to understand the subjects that influence a cervical cancer diagnosis.

## 3. Materials and Methods

The section mainly deals with the background research related to the research.

### 3.1. Predictions of Cancer Risk Factors

Cancer is the second leading cause of death globally, with about 9.6 million deaths in 2019. Cancer is caused when normal cells transform into tumor cells through a multistage process, mainly causing a malignant tumor [55]. However, cancer is more likely to respond to appropriate treatment with an increased chance of survival, less morbidity, and less-expensive therapy if identified earlier. Now, it is complex for a computer-aided diagnosis (CAD) system point of view to analyze the complex ecosystem created by screening and diagnosis methods. These complex issues worsen in numerous developing nations due to a lack of computing resources. For all the patients, who are skipping the routine screening, the major problems during diagnosis are identifying the best screening plan and estimating one's risk. The majority of the screening methods correlate with the physician's experience and subjective decision. To determine the riskiest group, one can apply the survey and reduce unnecessary screening. It helps to solve the cancer issues with a plan as per the cancer risk [56]. As per a World Health Organization new survey, cervical cancer has been the “4th greatest common type of cancer.” Once especially in comparison to other cancers, this is risky cancer. One such cancer is caused by being infected first alongside the HPV virus [57]. Many scientists discovered that the HPV viral infection is primarily transferred via sexual intercourse. There are many various varieties of HPVs, and cancer has been prompted by category sixteen and pattern 18. These are considered the highest HPVs because they cause cancer cell tissues in the area, so category six and category 11 have been considered significant HPVs because they cause cystitis on the surface [58].

Moreover, it has been found that an efficient and effective detection algorithm was a neural network in the past. The researchers described a TL regularization approach for different linear models, presenting its suitability in various contexts. Positive results have been gathered from this experiment. Other techniques used in cancer detection have been explored, like hierarchical clustering, ANN, and improved genetic algorithms. The authors [59] have performed classification on the cancer dataset, and the results have shown that performance varies between eighty and ninety percent approx. In 2016, the authors [60] had used different data mining techniques and classifiers to predict heart diseases. The researchers have presented the range of performance parameters between forty-five and ninety-nine percent approx. In 2017, the authors [61] did a comparative analysis of different machine learning models utilized for the early detection of heart disease.

### 3.2. Machine Learning Methods

It is a subfield of artificial intelligence (AI) that employs a diverse variety of measurable, statistical inference, and advancement strategies to assist machines in “knowing and understanding” from previous simulation models and comprehending complicated conceptual designs from tremendous, noisy, and complex statistical surveying [62]. Such capacity is helpful for medical applications that rely on complex proteomic and genotype estimate methodologies. Consequently, intelligence is routinely employed to detect and predict cancerous progression. Machine learning methods have increasingly been designed to estimate and forecast cancer [62].

#### 3.2.1. Support Vector Machines

The goal of the model is to find a higher dimensional venue in the *N*-dimensional area (where *N* represents the total of characteristics that characterize the datasets). Multiple hyperplanes might be used to describe them, but we want to find one with the most significant margin (distance between data points of both classes). Once it is accomplished, future measured values will be able to reinforce and categorized with increased confidence. SVM method creates a hyperplane in a relatively high or infinite space area, which helps in the data categorization process, regression, and other activities, i.e., extracting features and filtering [63].

The hyperplane with the longest distance towards the closest training stage of any category (as such production requires) achieves a better solution because the relatively large the percentage, the reduced the classifier's generalization error message, as described in

(1) $$\begin{array}{c} \left(X_{1},Y_{1}\right)\cdots \left(X_{n},Y_{n}\right), \end{array}$$

where *n* points and *X* and *Y* represent the class, *W* represents the normal vector, and *b* represents the parameter offset of the hyperplane. A hyperplane can be defined as described in

(2) $$\begin{array}{c} W^{T}\left(x-b\right)=0. \end{array}$$

#### 3.2.2. Decision Tree

DT is a type of nonsupervised learning technique that is commonly utilized for regression and classification problems. The aim is to expand a predictive model of the prediction error using standard decision rules and advanced analytic features [64]. A tree is an example of a fractional estimate. It is represented using the sum of product (SOP) method. Disjunctive normal structure is another name for SOP. So each division out from a massive tree root to just a subtree with the identical class is just a conjunction of attributes, and various branches terminating in that class establish a discontinuity. An entropy *E* can be represented as Equation (3). *E* represents entropy, *s* means samples, *Py* represents the probability of yes, *Pn* represents no, and *n* represents the number of samples.

(3) $$\begin{array}{c} E\left(s\right)=\overset{n}{\underset{k=0}{\sum }}\left(\begin{array}{c} n\\ k \end{array}\right)-Py*\log2Pn. \end{array}$$

#### 3.2.3. Random Forest

RF is a regression and classification tree-based ensemble learning algorithm. A bootstrap specimen size is used to train each tree, and perhaps optimum solution factors for each separation are chosen from a randomly selected subset of all elements. For regression and classification challenges, the selection processes are distinct. The Gini coefficient was used in the first case, while variance decrease was used in the second case. The RF's multilateral forecasting has been determined for regression and classification by calculating a majority of votes or an average [65]. The regression method might choose to get a binary result, allowing for probabilistic prediction comparable to regression analysis. The information gain for random forest can be calculated as defined in Equation (4), where *T* represents the target variable, *X* represents the feature set to be split, and Gain (*T*, *X*) represents the entropy value after dividing the data feature set *X*.

(4) $$\begin{array}{c} \text{Gain}\left(T,X\right)=\text{Entropy}\left(T\right)-\text{Entropy}\left(T,X\right). \end{array}$$

#### 3.2.4. Boruta Algorithm

The Boruta method was designed to represent all significant features within a classification model and therefore is designated after a deity of the forest through Slavic mythical. The primary idea behind this method is to use statistical procedures and multiple continuous runs of RFs to evaluate the significance of authentic predictors to arbitrary, as such edge factors. So every run doubles the number of predictors by duplicating them [65]. The shadow explanatory variable model is generated by removing redundant the actual values all over findings, destroying the connection with the results. The different evaluation principles have been accumulated. Compared to a random forest algorithm mainly learned on the enlarged given dataset, a quantitative test has been conducted for every complex variable; try to reach its significance to the sum of the entire shadow explanatory variable's maximum values.  Algorithm 1 shows the working of Boruta analysis [30, 31].

### 3.3. Problem Formulation and Proposed Model

It is assumed that coefficients can represent the model of cervical detection. The key objective can be understood to be a task(s) of finding an appropriate mathematical model that can be used for cervical cancer causal analysis and mathematically modeling.

There are two tasks involved in finding the changes in the set of variables (independent causal variables (*X*_1_, *X*_2_ ⋯ *X*_*i*_) or single independent variable concerning the influential variable (dependent variable *f*(*y*)) that leads to the development of cervical cancer in a subject. Both types of variables share the same vector space model. For a given task (*T*)⟶{{ *X*_1_, *X*_2_}, *Y*}, the mathematical relationship between these variables is represented by:

(5) $$\begin{array}{c} \left(T\right)⟶f\left(y\right)=\left({\text{Coff}}_{1}*X_{1}+{\text{Coff}}_{2}*X_{2}+{\text{Coff}}_{3}*X_{3}\cdots +{\text{Coff}}_{n}*X_{n},+C\right), \end{array}$$

where *X*_*i*_ is the set of cervical risk indicators, *f*(*y*) represents the effect that has happened due to *X*_*i*_, and Coff_1_ represents the cancer coefficient. We have created a variable, “cervical cancer,” which will be calculated by

(6) $$\begin{array}{c} \text{CervicalCancer}=\left[\text{Hinselman}+\text{Schiller}+\text{Citology}+\text{Biopsy}\right]. \end{array}$$

This research proposed an efficient feature selection and prediction model for cervical cancer datasets using Boruta analysis and SVM method to deal with existing challenges in cervical cancer prediction. A Boruta analysis method is used. It is improved from of random forest method and mainly discovers feature subsets from the data source that are significant to assign classification activity. The proposed model's primary aim is to determine the importance of cervical cancer screening factors for classifying high-risk patients depending on the findings. Data preprocessing phase plays an essential role in machine learning research because any missing value can affect the entire results. The validity of the data and the essential details that can be extracted significantly influence our model's potential to gain knowledge; thus, users must preprocess our statistics before supplying them to the proposed model.

## 4. Experiments and Analysis

This section presents the experimental findings and related consequences and discusses the proposed method's effectiveness over existing methods. This section evaluates numerous practical test parameters for the cervical cancer dataset and compares them with existing ML methods and the proposed methods.

### 4.1. Dataset Characteristics

The dataset consists of 36 attributes representing risk in terms of cervical cancer. Out of these 36 attributes, four attributes are categorical. The values of the categorical attributes are the outcome of the medical tests that have been conducted to verify the clinical finding on cervical cancer. The Hinselmann's test or the colposcopy test is done to check if the lesions are cancerous or not. In Schiller's test, a part of the body under observation is painted with a solution to investigate the malignant nature of the body part. The cytology test helps ascertain if there is some cancerous fluid in a body part. A complete biopsy is done when most of the standard clinical test options have been exhausted, and only a cut or biopsy can reveal the person's state of health about cancer, as described in Figure 1. Primary risk variables in constructing a cervical cancer forecasting model include using contraceptive pills, drinking, having many sex partners, and other body parameters.

In summary, the dataset consists of information about lifestyle habits such as smoking, information regarding the sexual behavior of the persons, and, last but not least, about the outcome of the medical tests. It can be observed that the attributes age, number of sexual partners (NSP), HC, and HCY have a correct level of variation, and other attributes' values do deviate from their mean values. It is because most of these values are Boolean in type. The dataset had a lot of empty values, which requires a missing values' treatment using the mean and median method.

### 4.2. Results and Hypothesis

Various machine learning-based models, random forest, SVM, decision tree, and Boruta method have been implemented in Python programming under an anaconda environment.

Table 4 represents the relationship between parameters mainly used for the hypothesis: the dependent parameters and their possible predictors.

#### 4.2.1. Confusion Matrix

It is a means of expressing the effectiveness of a classifier's technique. Once individuals have an inequity number of incidents for each class and when individuals have more than two classes in the data source, a classification performance can be vague (Figure 2).

#### 4.2.2. Experimental Investigation 1

**Hypothesis 1 .**

Does weight (WT) depend on other parameters or have strong relationships with others.

Interpretation of model 1: Figure 3 shows that the correlation coefficient (coef) varies from 9.936*e*-17 to -0.00989 for different parameters. The coefficient from 0.1 to 0.5 is considered a weak value, and more than 0.5 is considered a substantial value. The *p* values show that all parameters are significant as the *p* value is (*p* ≤ 0.01) for all the variables except in the case of BP-dia, which has a value of 0.99. Moreover, all the parameters have low errors. The intercept has a positive value of 9.93. The data values mainly focus on the mean as SM and VF coefficient values are negative. The total frequency of the findings revealed large tails, indicating that there is no association between dependent class and even the strongest predictor's class of prototype (as described in model 1).

#### 4.2.3. Experimental Investigation 2

**Hypothesis 2 .**

The value of visceral fat is just a combination of other parameters that directly correlate with others and predictions and verification.

Interpretation of model 2: in Figure 4, the values of coef are less than 0.5, which shows a week selection. Also, the standard errors turn out to be close to zero in most cases. At the same time, negative coefficients attribute to it. The *p* values are ≤0.01, suggesting all the variables' significance and importance. The intercept is positive. The dataset depicts a low level of skewness (shapes are not symmetrical), but massive tails are observed. All these factors fail to acquire the correct coef value.

#### 4.2.4. Experimental Investigation 3

**Hypothesis 3 .**

This hypothesis mainly considers body age (BA) data and verifies cancer-based on body age. Is the BA a consequence of all the other parameters, or does it have a strong link?

Interpretation of model 3: Figure 5 shows that the *p* value for all variables is ≤0.01, and it describes that all variables are significant, and this reason stresses including all the significant variables in model 3. The two variables negatively correlate with BA, BMI, and BPsys, whereas all left variables positively correlate with BA. A significant difference was found between the fitted and actual variables' values as they have low standard error except for BDA. The Coef values indicate that the model is not a good fit. The model fails to explain the relationship between BA and other variables.

#### 4.2.5. Experimental Investigation 4

**Hypothesis 4 .**

this hypothesis mainly considers the blood pressure systolic (BpIsys) to predict cancer in the body. A BPSys parameter can be used as a function and represent the combination of other parameters with a strong relationship with the other parameters.

Interpretation of model 4: almost all factors have *p* values of nil, as shown in Figure 6, which indicates that they are significant and should be incorporated into the equation. Variables BA and BPdia show a minimal negative correlation with the dependent variables (BPSys), whereas a positive correlation is seen with the rest. As a result, we can imply that the regression method had difficulty finding a good fit. It performed pretty finding a good fit as the Coef value (0.754), but the model needs to be rejected with an onset of a better model. Compared with the first model (VF), this model suggests BPSys cannot be a function of all other variables 1.2. The Durbin-Watson test indicates that a high amount of overlap is not desirable.

#### 4.2.6. Experimental Investigation 5

**Hypothesis 5 .**

This hypothesis mainly considers the skeleton muscle (SM). This hypothesis verifies how the SM parameters can be utilized as a cumulative function of other factors with a strong relationship with the numerous parameters.

Interpretation of model 5: the coef is 0.78, which is lower than its VF method designed during the first experiment research. According to the Durbin-Watson results shown in Figure 7, the system has a moderate correlation, indicating that it is just not fit.

#### 4.2.7. Experimental Investigation 6

Hypothesis: in hypothesis 6, we mainly consider the machine learning models. Can the leering machine model with mathematical equations predict cervical cancers accurately? In this experimental investigation, we consider all the hypotheses from 1 to 6 and apply them to various machine learning methods.

Interpretation of model 6: this model utilizes machine learning methods, i.e., random forest, SVM, and decision tree methods. The original data is arbitrarily divided into training and testing pairs to ensure the results obtained are accurate that can be used to create forecasting models. Inside this research work, 70% of the dataset has been used for training, while 30% is used for test results.

The random forest variable's design is directed at the classification method. The overall percentage of vertices inside the RF (the data variable ntree) has been set to 300. Inside the RF method, the total number of trees which will grow appears to be ntree. We must verify that for almost every source sequence predicted at least very few mins max, the ntree should not be set to a restricted fraction. The study results again for the random forest approach, as shown in Figure 8. In aspects of constructing a predictive model, sixteen samplings have been currently examined for accurate test data. The confusion matrix can have been examined when executing the prediction on the dataset. A confusion matrix can be seen in Figure 6. The confusion matrix will be used to determine how efficient the classifier has been as a prediction. The algorithm anticipated that 7 out of the total eight observations again for normal data sample would be “normal,” although the left standing data sample that was only 1 sample data would be because of cancer. The obtained measurements for SVM approaches are shown in Figure 9.

The precision of the decision tree classifier achieved is greater than 86 percent, which may be appropriate throughout many implementations. In trying to predict cervical cancer, random forest (RF) methods now have one of the highest accuracy appearances.  Figure 10 shows the experimental results for the decision tree methods.  Figure 11 shows the experimental results for the Boruta analysis methods.

### 4.3. Boruta Analysis and Causal Mathematical Modeling Results

In this section, analyses of all the indicators of cancer are done so that only those variables are used in building an equation model that is useful in detecting cervical cancer. In other words, in this section, the elimination of those variables is done, which does not mathematically correlate to the medical biopsy test. For this purpose, correlation and Boruta importance analysis is done. It is a well-known fact that correlation does not mean a causal relationship between the variables. However, it gives an idea of how strong and weak the relationship is between the variables. Lower correlation values mean the two variables do not have much impact on each other. The Boruta technique evaluated variable importance by swapping predictor qualities and combining them only with initial predictive variables before constructing a random forest upon that fully integrated dataset. After that, we will compare the independent dataset to the randomly selected samples to predict their significance and select something with a higher significance than the randomly selected factors.

According to this graphical analysis (Figure 12), the variables (a) Schiller, (b) Hinselmann, and (c) Cytology have been the most helpful in cervical cancer prediction. Another option for selecting the features is to consider the factors used the most by so many machine learning techniques just to be substantial. Machine learning algorithms first discover the relationship among *Xs* and *Ys*, and then, depending on the learning, numerous machine learning methods may utilize multiple parameters to differing extents. As a result, factors that worked well in a tree-based method like modification or destruction may be undervalued in a linear interpolation model.

As a result, all the factors must be perfectly acceptable for all methodologies. Using an application in a number in ML to select selected features can improve classification performance.  Figure 13 shows the Boruta analysis for cervical cancer prediction. It is an algorithm that identifies the importance of the variables for the given categorical variable. This algorithm covers the minimum-optimal feature selection and the all relevant selection strategy. It provides output in terms of three categories, i.e., the most critical variables and tentatively that are significant during evaluation, and the third category is the rejected features or variables. This algorithm is a wrapper around the random forest algorithm, and its sole purpose is to help select essential variables for further analysis.

Figures 14 and 15 show the details of cervical cancer classes and types (age-based). The cervical cancer classes can be classified into five categories (0, 1, 2, 3, 4, and 5). A correlation histogram showed that two considerations had no other details once all the missing data were filled in (a) sexually transmitted diseases: cervical condylomatosis and (b) sexually transmitted infections (STIs): AIDS. We removed these variables from the dataset and used a comparison heatmap on how each one is connected to the attribute value “tissue sample.” Boruta's scaling characteristics are the number of characteristics (destroyed) and the collection of instances (correct). So every edge just on the leftmost column refers to a set of particles of the same number of components, so each edge on the top right equates to several characteristics with almost the same number of features. It is worth noting that scalability is sequential concerning the number of features and not so much in terms of the total quantity of particles.

Table 5 represents the results of the cervical indicators for Boruta analysis and correlation analysis. From both kinds of feature analysis, it is clear that “Schiller,” “Hinselmann_1,” and “Cytology” (medical test) had the highest correlation with biopsy. This means that most medical tests clinically support evidence for cervical cancer. Table 4 gives the output of both these analyses. Logically, some of the attributes out of 36 attributes need to drop. Based on the UCI cervical cancer database, a combination of eighteen characteristics and four diagnostic testing findings are significant for constructing a causality assessment report on cervical cancer. A more profound analysis shows both the methods have found those essential variables: number of sexual partners, Dx: cancer, Dx, STDs: vulvoperineal_condy_lomatosis, STD: condy_lomatosis, hormonal contraceptives (years) are essential.

Hence, it is logical to construct a causal analysis based on these variables. The correlation confirmed that this group of variables is strongly associated. The Boruta algorithm ensures that these variables are significant and vital for further analysis. The analysis confirms the correlation in a few pairs [65]. It is challenging to cover all the dependent and prediction variables due to low correlation values. Then, the section builds a hypothesis around these variables to identify which variable can act as a dependent variable to predict the changes in the dynamics of cervical analysis. Hence, only those variables are used for the subsequent analysis that affects each other and helps predict cervical cancer. Thus, a cervical cancer causal analysis would be formed or nullified by proving a null hypothesis test value. Table 5 gives a set of hypotheses. Multiple performance metrics have been used to enhance the accuracy of clinical overall result forecasting.

Figure 16 shows results for Boruta analysis vs. existing methods. The machine learning methods have been calculated for random forest, SVM, decision tree, and Boruta analysis on cancer (i.e., cervical cancer) dataset. This research applied ML techniques (random forest, decision tree, SVM, and Boruta analysis) [32] towards cervical cancer prediction and helps in diagnosis to underline the necessity of model development with evidence, considering all the outstanding selected data features such as data cleansing, substituting missing values, and applying a feature extraction approach to increase implications predictions efficiency. This research also utilized ML models to predict the cervical cancer detection risk factors, bearing in mind all the information only within the dataset by substituting variables in the columns by their mean and deleting just the portions with a missing value.

The forecasting results of the models' coefficient values are near 1, indicating that none of them have reached a high degree of efficiency. In each of the scenarios developed, the diverse range of skills has a substantial effect. Even as *t*-test data demonstrated, this correlation between the dependency and independent factors can be completely ruled out. Different scenarios also have expected to be high over 0.76, and the other has a frequency of 0.789 results. The value of cumulative impacts can be calculated as follows:

(7) $$\begin{array}{c} y\left(\text{VFx}\right)=\left[\left(0.0138*\left(\text{BA}\right)\right)+\left(0.0811*\left(\text{BDA}\right)\right)-\left(0.0112*\left(\text{WT}\right)\right)+\left(0.0128*\left(\text{BMI}\right)\right)—\left(0.0419*\left(\text{BPsys}\right)\right)—\left(0.0106*\left(\text{BPdia}\right)\right)+\left(0.0201*\left(\text{SMn}\right)+2.05e-14\right)\right]. \end{array}$$

The experimental values for cervical cancer forecasting using a machine learning algorithm are shown in Figure 16. The obtained Figure 16 measurements are shown for the random forest methodology (precision is 0.889, recall is 0.875, *F*1 score is 0.757, and support is 0.745). In contrast, the obtained measurements are shown for the decision tree technique (precision is 0.8657, recall is 0.865, *F*1 score is 0.718, and support is 0.7256). The casual analysis works on the regression process that confirms the statistical relationship between cervical cancer parameters. The results show that “Schiller,” “Hinselmann_1,” and “Cytology” are the main parameters predicting cervical cancer. When performing superficial root investigation with various parameters, a detailed examination and exploitation of six distinct hypotheses reveal visceral fat represents a healthcare indication and might be a strong predictor of anyone's health. This parameter indicates that since the rates of other factors include personage, body type, BMI, BP, the metabolism rate, and other essential parameters can represent the correct value of visceral fat. This approach also gives information just on the beginning of medical conditions. The method is verified using multiple measures, including statistical Boruta analysis and correlation, on various machine learning methods.

## 5. Conclusion and Future Work

In this research, a mathematical machine learning-based model has been developed for analyzing various possibilities of cervical cancer. The prediction has been studied by using multiple eight body factors. This research work analyses cervical cancer and various risk factors contributing to its development. The authors view the statistical technologies, machine learning, and methodologies that can help detect cervical cancer after identifying the paper's research gaps. In addition, this research utilized SVM, random forest, decision tree, and Boruta investigation to create a few classification models. Optimum prospects have been investigated for the development and performance assessment of all modeling techniques. The accuracy and quality of all these methodologies have been analyzed in this article based on the data obtained. Overall, statistical Boruta analysis and random forest methods have performed reasonably well with accuracy, precision, and other parameters for identifying cervical cancer risk and type. The SVM machine learning model produces comparable findings (precision is 0.8456, recall is 0.812, *F*1 score is 0.684, and support is 0.717). At the same time, the Boruta analysis shows comparable findings (precision is 0.912, recall is 0.891, *F*1 score is 0.798, and support is 0.768). Compared to other machine learning-based algorithms, the experimental results suggest that Boruta analysis performed best.

Furthermore, this comprehensive evaluation of contouring efficiency may be used to analyze the diagnostic value of fully automated feature extraction in future work. Emerging technologies and methods should be stimulating in research to predict cervical cancer. We can work on socio-demographic factors such as the region of sample data selected and the level of education of that particular region. Educational institutions and schools can contribute to extending the awareness to families of the children they are teaching for their better healthcare.

## Figures and Tables

**Figure 1:** Variable distribution in the cervical cancer dataset.

**Figure 2:** Confusion matrix for random forest, SVM, and decision tree.

**Figure 3:** WF having a relationship with other variables.

**Figure 4:** Visceral fat (VF) having a relationship with other variables.

**Figure 5:** BA having a relationship with other variables.

**Figure 6:** BPSys having a relationship with other variables.

**Figure 7:** SM has a relationship with other variables.

**Figure 8:** Experimental results for the random forest method.

**Figure 9:** Experimental results for the SVM method.

**Figure 10:** Experimental results for decision methods.

**Figure 11:** Experimental results for Boruta analysis methods.

**Figure 12:** Boruta analysis based on selected features.

**Figure 13:** Boruta analysis based on all features.

**Figure 14:** Cervical cancer based on age.

**Figure 15:** Cervical cancer classes.

**Figure 16:** Experimental results for Boruta analysis vs. existing methods.

**Algorithm 1:** Boruta algorithm.

**Table 1:** Comparison of a research review on risk factors for cervical cancer.

Article	Risk factors discussed	Imported feature (age group)	Possible cancer types
[15]	Human papilloma-virus (HPV) infection	18-35	Cervical cancer, breast cancer
[16]	Sexual history	Under 18 and above	Carcinoma, cervical cancer
[17]	Smoking	All age groups	Lung, cervical, and breast cancer
[18]	Weakened immune system	30-60	Carcinoma, cervical cancer
[19]	Chlamydia infection	All age groups	Carcinoma, cervical cancer
[20]	Oral contraceptives do with a long period (birth control pills)	18-50	Cervical cancer, lung
[21]	Several full-term pregnancies	18-40	Cervical cancer, lung
[22]	First full-term pregnancy at a young age	25-60	Cervical cancer, lung
[23]	A diet deficient in fruits and veggies	22-56	Cervical cancer, lung
[24]	Smoking and HPV	11-60	Cervical cancer, lung
[25]	Use of pills (pregnancy)	22-45	Cervical cancer, lung
[26]	Early pregnancy, HPV	13-18	Cervical cancer, lung
[27]	HPV and weaker immunity	18-50	Cervical cancer, lung

**Table 2:** Review of cancer type based on no of features and age group.

Article	No of features selected	Imported feature (age group)	Possible cancer types
[33]	13 parameters	18-40	Cancer type 1 and type 2
[34]	10 parameters	20-50	Cervical cancer, lung cancer
[35]	12 parameters	18-55	Cervical cancer, skin cancer
[36]	10 parameters	18-45	Cervical cancer type 3
[37]	15 parameters	20-50	Cervical cancer, breast cancer
[38]	7 parameters	18-30	Cervical cancer, breast cancer
[39]	10 parameters	17-30	Cervical cancer, lung cancer
[40]	18 parameters	14-60	Cervical cancer, type 2 and 3
[41]	12 parameters	15-55	Cervical cancer, type 1

**Table 3:** Comparison of a research review based on machine learning methods.

Article	Technique utilizes	Type of cancer	Important feature discussed	Dataset used	Validation technique
[47]	Artificial neural network	Cancer in breast	Age and mammography results	Diagnostics data and pathological data	Crossvalidation 10-fold
[48]	Support vector machine	Cancer multiple myeloma	STAT1, BRCA1, and CCND1 CCNB1	Online UCI	Crossvalidation 20-fold validation
[49]	Random forest	Cervical cancer	Diet, eating habits, and BME	Clinical data	Crossvalidation 10-fold
[50]	BN methods	Lung cancer	BP, age, and other parameters	Kaggle online dataset	10-fold crossvalidation
[51]	SVM	Cervical cancer, breast cancer	Skin type, breast size, and skin color	Dataset from the hospital (China)	Clinical survey data
[52]	Boruta	Cervical cancer, lung and breast	Age, infection type	Clinical survey data	Crossvalidation
[53]	SVM with random forest	Cervical cancer, cancer in lungs	BME	UCI online dataset	10-fold crossvalidation
[54]	K-NN, SVM	Cervical cancer	Age and mammography results	UCI dataset	Crossvalidation 10-fold

**Table 4:** The hypothesis to find the relationship between the parameters.

S. no.	Hypothesis	
	Dependent parameter	Possible predictors
1	Sexual partners' frequency	Sexual partners' frequency, Dix: cancer, Dix, STDs: hormonal contraception via hormones (years) vulvoperinea_lcondy_lomatosis
2	Dix: cancer	Sexual partners' frequency, Dix: cancer, Dix, STDs: hormonal contraception via hormones (years) vulvoperinea_lcondy_lomatosis
3	STDs: vulvoperinea_lcondy_lomatosis	Sexual partners' frequency, Dix: cancer, Dix, STDs: hormonal contraception via hormones (years), vulvoperinea_lcondy_lomatosis
4	STDs: condy_lomatosis	Sexual partners' frequency, Dix: cancer, Dix, STDs: contraception via hormones (years), vulvoperinea_lcondy_lomatosis
5	Contraception via hormones (years)	Sexual partners' frequency, Dix: cancer, Dix, STDs: contraception via hormones (years), vulvoperinea_lcondy_lomatosis

**Table 5:** Cervical indicators results for Boruta analysis and correlation analysis.

S. no.	Cancer indicator	Boruta analysis	Correlation analysis
Number of sexual partners		√	√
1	Smoke	√	X
2	Smoke (years)	√	X
3	Smoke (packs)	√	X
4	Hormonal contraceptives (years)	√	X
5	IUD	√	X
6	IUD (years)	√	X
7	STD: number	√	X
8	STD: condylomatosis	√	X
9	STDs: vulvo-perineal condylomatosis	√	√
10	STD: syphilis	√	X
11	STD: time since the first diagnosis	√	X
12	STD: genital herpes	X	√
13	STD: HIV	X	√
14	STD: time since last diagnosis	√	X
15	Dx	√	√
16	Dx_cancer	√	√
17	Dx_HPV	√	√
18	Dx_CIN	√	X
19	Dx_CIN	X	√
20	Dx_CIN	X	√

## Data Availability

The data used to support the findings of this study are available from the corresponding author upon request.

## References

[1] Park Y. R., Kim Y. J., Ju W., Nam K., Kim S., Kim K. G. (2021). Comparison of machine and deep learning for the classification of cervical cancer based on cervicography images. *Scientific Reports*.

[2] Chang C. C., Cheng S. L., Lu C. J., Liao K. H. (2013). Prediction of recurrence in patients with cervical cancer using MARS and classification. *International Journal of Machine Learning and Computing*.

[3] Poongodi M., Hamdi V., Vijayakumar B. S., Rawal M., Maode An effective electronic, waste management solution, based on blockchain smart contract in 5G communities.

[4] Chu R. (2021). Risk stratification of early-stage cervical cancer with intermediate-risk factors: model development and validation based on machine learning algorithm. *The Oncologist*.

[5] Charoenkwan P., Shoombuatong W., Nantasupha C., Muangmool T., Suprasert P., Charoenkwan K. (2021). IPMI: machine learning-aided identification of parametrial invasion in women with early-stage cervical cancer. *Diagnostics*.

[6] Zixian Z., Xuning L., Zhixiang L., Hongqiang H. (2021). Outburst prediction and influencing factors analysis based on Boruta-Apriori and BO-SVM algorithms. *Journal of Intelligent Fuzzy Systems*.

[7] Varalakshmi A., Lakshmi A., Swetha A., Rahema M. A comparative analysis of machine and deep learning models for cervical cancer classification.

[8] Luo W. (2021). Predicting cervical cancer outcomes: statistics, images, and machine learning. *Frontiers in Artificial Intelligence*.

[9] Poongodi M., Vijayakumar V., Chilamkurti N. (2020). Bitcoin price prediction using ARIMA model. *International Journal of Internet Technology and Secured Transactions*.

[10] Jajodia A., Gupta A., Prosch H. (2021). Combination of radiomics and machine learning with diffusion-weighted MR imaging for clinical outcome prognostication in cervical cancer. *Tomography*.

[11] Patil M. M. (2021). The machine learning algorithm for prediction of risk factors of cervical cancer. *International Journal for Research in Applied Science and Engineering Technology*.

[12] Kumar P., Kumar R., Srivastava G. (2021). PPSF: a privacy-preserving and secure framework using blockchain-based machine-learning for IoT-driven smart cities. *IEEE Transactions on Network Science and Engineering*.

[13] Poongodi M., Bose S. (2015). Detection and prevention system towards the truth of convergence on decision using Aumann agreement theorem. *Procedia Computer Science*.

[14] Ding D., Lang T., Zou D. (2021). Machine learning-based prediction of survival prognosis in cervical cancer. *BMC Bioinformatics*.

[15] Guo C., Wang J., Wang Y. (2021). Novel artificial intelligence machine learning approaches to precisely predict survival and site-specific recurrence in cervical cancer: a multi-institutional study. *Translational Oncology*.

[16] Poongodi M., Vijayakumar V., Rawal B. (2019). Recommendation model based on trust relations & user credibility. *Journal of Intelligent & Fuzzy Systems*.

[17] Yin Q. The application of machine learning in cervical cancer prediction.

[18] Singh K., Lilhore U. K., Agrawal N. (2017). Survey on different tumour detection methods from MR images. *International Journal of Scientific Research in Computer Science, Engineering and Information Technology 2*.

[19] Akter L., Ferdib-Al-Islam M. M., Islam M. S., Al-Rakhami M. R., Haque (2021). Prediction of cervical cancer from behavior risk using machine learning techniques. *SN Computer Science*.

[20] Gupta A., Anand A., Hasija Y. Recall-based machine learning approach for early detection of cervical cancer.

[21] Prianka C., Kavida B. (2021). Cervical cancer cell prediction using machine learning classification algorithms. *Engineering and Scientific International Journal*.

[22] Jahan S., Islam M. D. S., Islam L. (2021). Automated invasive cervical cancer disease detection at early stage through suitable machine learning model. *SN Applied Sciences*.

[23] Arora A., Tripathi, Bhan Classification of cervical cancer detection using machine learning algorithms.

[24] Iwendi O., Allen A. R. Enhanced security technique for wireless sensor network nodes.

[25] Weegar R., Sundström K. (2020). Using machine learning for predicting cervical cancer from Swedish electronic health records by mining hierarchical representations. *PLoS One*.

[26] Lu J., Song E., Ghoneim A., Alrashoud M. (2020). Machine learning for assisting cervical cancer diagnosis: an ensemble approach. *Future Generation Computer Systems*.

[27] Poongodi M., Bose S. Design of intrusion detection and prevention system (IDPs) using DGSOTFC in collaborative protection networks.

[28] Hassan A., Prasad D., Khurana M., Lilhore U. K, Simaiya S. (2021). Integration of internet of things (IoT) in health care industry: an overview of benefits, challenges, and applications. *Data Science and Innovations for Intelligent Systems*.

[29] Ramesh T. R., Lilhore U. K., Poongodi M., Simaiya S., Kaur A., Hamdi M. (2022). Preditive analysis of heart diseases with machine learning approaches. *Malaysian Journal of Computer Science*.

[30] Ramzan Z., Hassan M. A., Asif H. M. S., Farooq A. (2020). A machine learning-based self-risk assessment technique for cervical cancer. *Current Bioinformatics*.

[31] Ghoneim A., Muhammad G., Hossain M. S. (2020). Cervical cancer classification using convolutional neural networks and extreme learning machines. *Future Generation Computer Systems*.

[32] Kaur A., Mann K. S. (2017). Skeletal bone age assessment using neural network. *International Journal Of Research In Electronics And Computer Engineering*.

[33] Singh S. K., Goyal A. (2020). Performance analysis of machine learning algorithms for cervical cancer detection. *International Journal of Healthcare Information Systems and Informatics*.

[34] Kim S., Lee S., Choi C. H. (2021). Machine learning models to predict survival outcomes according to the surgical approach of primary radical hysterectomy in patients with early cervical cancer. *Cancers*.

[35] Trivedi N. K., Simaiya S., Lilhore U. K., Sharma S. K. (2021). COVID-19 pandemic: role of machine learning & deep learning methods in diagnosis. *International Journal of Current Research and Review*.

[36] Lilhore U. K., Simaiya S., Prasad D., Guleria K. (2020). A hybrid tumour detection and classification based on machine learning. *Journal of Computational and Theoretical Nanoscience*.

[37] Lilhore U. K., Simaiya S., Guleria K., Prasad D. (2020). An efficient load balancing method by using machine learning-based VM distribution and dynamic resource mapping. *Journal of Computational and Theoretical Nanoscience*.

[38] Patel D. T. S. (2018). A cross sectional study to estimate delay in diagnosis and treatment of tuberculosis (TB) among patients attending urban health centre in an urban slum area. *Public Health Review: International Journal of Public Health Research*.

[39] Guleria K., Sharma A., Lilhore U. K., Prasad D. (2020). Breast cancer prediction and classification using supervised learning techniques. *Journal of Computational and Theoretical Nanoscience*.

[40] Gupta L., Edelen A., Neveu N., Mishra A., Mayes C., Kim Y. K. (2021). Improving surrogate model accuracy for the LCLS-II injector frontend using convolutional neural networks and transfer learning. *Machine Learning: Science and Technology*.

[41] Fei D. Y., Almasiri O., Rafig A. (2020). Skin cancer detection using support vector machine learning classification based on particle swarm optimization capabilities. *Transactions on Machine Learning and Artificial Intelligence*.

[42] Liew X. Y., Hameed N., Clos J. (2021). An investigation of XGBoost-based algorithm for breast cancer classification. *Machine Learning with Applications*.

[43] Ali M. S., Miah M. S., Haque J., Rahman M. M., Islam M. K. (2021). An enhanced technique of skin cancer classification using a deep convolutional neural network with transfer learning models. *Machine Learning with Applications*.

[44] Park Y. (2021). Classification of cervical cancer using deep learning and machine learning approach.

[45] Abadi A. M., Departnment D. U., Wustqa N., Nurhayadi (2019). Diagnosis of brain cancer using radial basis function neural network with singular value decomposition method. *International Journal of Machine Learning and Computing*.

[46] Wu N., Jastrzębski S., Park J., Moy L., Cho K., Geras K. J. (2020). Improving the ability of deep neural networks to use information from multiple views in breast cancer screening. *The Proceedings of Machine Learning Research*.

[47] Dataset Dataset. https://archive.ics.uci.edu/ml/datasets/Cervical+cancer+%28Risk+Factors%29.

[48] Lilhore U. K., Imoize A. L., Lee C.-C. (2022). Enhanced convolutional neural network model for cassava leaf disease identification and classification. *Mathematics*.

[49] Zhou Z., Maquilan G. M., Thomas K. (2020). Quantitative PET imaging and clinical parameters as predictive factors, for patients with cervical- carcinoma: implications of a prediction model generated using multi-objective support vector machine learning. *Technology in Cancer Research & Treatment*.

[50] Kapil S., Lilhore U. K., Agarwal N. (2018). An improved data reduction technique based on KNN & NB with hybrid selection method for effective software bugs triage. *International Journal of Scientific Research in Computer Science, Engineering and Information Technology*.

[51] Kaushik M., Chandra Joshi R., Kushwah A. S. (2021). Cytokine gene variants and socio-demographic characteristics as predictors of cervical cancer: a machine learning approach. *Computers in Biology and Medicine*.

[52] Trivedi N. K., Simaiya S., Lilhore U. K., Sharma S. K. (2020). An efficient credit card fraud detection model based on machine learning methods. *International Journal of Advanced Science and Technology*.

[53] Kaur A., Mann K. S. (2017). A novel framework for cloud-based bone age assessment integration system: review and analysis. *International Journal of Computational Engineering Research*.

[54] Sharma S., Kumar U., Lilhore S. K., Simaiya N. K., Trivedi (2021). An improved random forest algorithm for predicting the COVID-19 pandemic patient health. *Annals of the Romanian Society for Cell Biology*.

[55] Iwendi S., Khan J. H., Anajemba A. K., Bashir F., Noor (2020). Realizing an efficient IoMT-assisted patient diet recommendation system through machine learning model. *IEEE Access*.

[56] Kaur A., Mann K. S. (2018). Segmenting bone parts for bone age assessment using point distribution model and contour modeling. *Journal of Physics: Conference Series*.

[57] Patil V., Lilhore U. K. (2018). A survey on different data mining & machine learning methods for credit card fraud detection. *International Journal of Scientific Research in Computer Science, Engineering and Information Technology*.

[58] Kaur A., Mann K. S. (2019). Hybrid classifier for bone age assessment.

[59] Dhanamjayulu C., Nizhal U. N., Maddikunta P. K. R., Gadekallu T. R., Iwendi C. (2021). Identification of malnutrition and prediction of BMI from facial images using real-time image processing and machine learning. *IET Image Process*.

[60] Iwendi (2020). Sanitization: a semantic privacy-preserving framework for unstructured medical datasets. *Journal: Computer Communications*.

[61] Abbas S., Jalil Z., Javed A. R. (2021). BCD-WERT: a novel approach for breast cancer detection using whale optimization-based efficient features and extremely randomized tree algorithm. *PeerJ Computer Science*.

[62] Simaiya S., Lilhore U. K., Prasad D., Verma D. K. (2021). MRI brain tumour detection & image segmentation by hybrid hierarchical K-means clustering with FCM based machine learning model. *Annals of the Romanian Society for Cell Biology*.

[63] Kaur A., Khurana M., Kukreja V., Jindal P., Geetanjali Skeletal growth assessment using segmented middle phalanx with active shape modelling.

[64] Tiwari S., Lilhore U., Singh A. (2018). Artificial neural network and genetic clustering based robust intrusion detection system. *International Journal of Computer Applications*.

[65] Kaur A., Mann K. S. (2018). Bone age classification using SVM' international journal of engineering science invention. *International Journal of Engineering Science Invention*.

